The article "Consequence of Two Protocols of Social Defeat Stress on Nicotine-Induced Psychomotor Effects in Mice" was published in 2019. Journal: Biomed Res Int.

# Consequence of Two Protocols of Social Defeat Stress on Nicotine-Induced Psychomotor Effects in Mice

**DOI:** 10.1155/2019/5404251

**Published:** 2019-04-24

**Authors:** Liz Paola Domingues, Bruno de Brito Antonio, Maria Gabriela Menezes de Oliveira, Isabel Marian Hartmann de Quadros

**Affiliations:** Departamento de Psicobiologia, Universidade Federal de São Paulo, Brazil

## Abstract

Exposure to stress may contribute to enhanced vulnerability to drug use disorders, by altering sensitivity to drug-related reward and psychomotor effects. This study aimed to characterize the psychomotor effects of nicotine administration and then investigate the consequences of two types of repeated social defeat stress (episodic and continuous) on nicotine-induced psychomotor effects in mice. Adult male Swiss mice were treated for 13 days with daily injections of nicotine (0.1, 0.4, or 1.0 mg/kg, s.c.) and received saline and nicotine challenges (0, 0.1 and 0.4 mg/kg) after a withdrawal period. Dose-dependent effects were observed in locomotor response to nicotine, with trends for locomotor stimulation after intermittent (but not acute) administration of 0.1 mg/kg. Higher nicotine doses caused acute locomotor suppression (0.4 and 1.0 mg/kg) and tolerance after intermittent administration (0.4 mg/kg dose). In separate cohorts, experimental mice were daily defeated by aggressive mice, using the resident-intruder model, for 10 days. After brief confrontations, intruders returned to their home cage (episodic stress) or were continuously exposed to the aggressive resident for 24 h (continuous stress), until the following defeat. After the 10-day stress protocol, mice received saline and nicotine challenges (0 and 0.1 mg/kg, s.c.) in locomotor tests. Mice were also tested for methamphetamine-induced locomotor response (1.0 mg/kg, i.p.). Both defeat protocols induced short-term locomotor suppression (24h after stress), which was further suppressed by nicotine only in mice exposed to continuous defeat stress. Ten days after stress, locomotor behavior was no longer suppressed in defeated mice of either stress protocol. Mice exposed to continuous defeat stress showed a reduced stimulant response to methamphetamine, 12 days after termination of stress. Our findings indicate that exposure to continuous defeat stress facilitates nicotine-induced locomotor suppression shortly after stress and reduces methamphetamine-induced stimulation in the long term.

## 1. Introduction

According to the World Health Organization [1], 21% of the adult population smokes worldwide. Smoking is associated with 90% of lung cancer cases and is a significant risk factor for other cancers, strokes, heart attacks, and chronic obstructive pulmonary disease [2]. For this reason, smoking is considered the leading cause of preventable death in the world [1, 3]. Out of several substances found in tobacco-derived products, nicotine is the principal psychotropic compound associated with reinforcing smoking behavior and promoting tobacco use disorders and dependence [3, 4].

Similarly to other addictive substances such as alcohol, cocaine, and amphetamines, nicotine promotes reinforcing effects and locomotor stimulation by activation of dopamine brain reward systems [5–8]. Chronic, repeated exposure to nicotine and other drugs may potentiate drug-induced increases in accumbal dopamine, attributing increased salience to the drug and drug-related stimuli [7, 9–11]. Neural and behavioral responses to the drug would then contribute to the development and maintenance of drug addiction [10–12].

Stress promotes enhanced vulnerability to drug use disorders, from initial use to dependence and relapse [13–15], as corroborated in animal models [16, 17]. In animal models, exposure to stress may also sensitize dopamine reward systems, rendering animals more sensitive to drug effects and reward [11, 17–20]. However, outcomes may differ according to characteristics of the stressor, duration of stress exposure, and stress protocols. For example, there is evidence that chronic restraint stress potentiates the stimulant effects of nicotine in rats [21], what is not observed after social isolation stress [22]. Rats exposed to chronic mild stress also presented cross-sensitization to nicotine locomotor effects, as well as increased nicotine seeking in a self-administration protocol [23]. However, Al-Hasani et al. (2013) [24] reported that chronic mild stress failed to interfere with conditioned reward to nicotine, using a conditioned place preference model in mice.

Repeated exposure to brief episodes of social defeat stress potentiates psychostimulant-induced locomotor stimulation, the acquisition rate, and motivation to self-administer cocaine and amphetamine [16, 25–27]. Repeated social defeat stress also facilitates the acquisition of cocaine-induced conditioned place preference in mice [28]. However, different protocols of social defeat stress seem to promote differential impacts on accumbal dopamine function and drug-related behaviors [18]. On one hand, brief episodes of social defeat reliably induce a sensitized dopamine response, locomotor cross-sensitization, and increased psychostimulant self-administration (e.g., [18, 27]). On the other hand, when defeat episodes are followed by cohabitation with the aggressor (“continuous” defeat, subordination stress), rats show blunted dopamine levels, tolerance to cocaine stimulation, and reduced cocaine intake [18]. Nonetheless, continuous defeat stress in mice has also been shown to promote increased dopamine neuronal firing in the VTA, and increased neuroplasticity in the accumbens [29, 30]. Thus, while chronic social stress consistently impacts brain reward function and plasticity, the precise mechanisms and outcomes may differ according to specific procedures, species, duration of stress exposure, etc.

Furthermore, it is also interesting that the consequences of social defeat stress seem to vary according to the drug tested. Differently from psychostimulants, there was no major impact of episodic defeats on heroin intake [31], and effects on alcohol reward are quite variable (e.g., [32, 33]) and may depend on the intensity of the aggressive confrontations [34]. The present study investigated the consequences of exposure to two types of repeated social defeat stress (episodic and continuous) on nicotine-induced psychomotor effects in mice. We hypothesized that repeated episodic stress would enhance nicotine psychomotor effects, while continuous stress would blunt nicotine's effects, similarly to what was reported for cocaine in rats [18].

## 2. Material and Methods

### 2.1. Subjects

Male Swiss mice (60 days old) were obtained from the Center for Experimental Models (CEDEME) at the Universidade Federal de São Paulo (UNIFESP, São Paulo, Brazil). Mice were individually housed in plastic cages (30 × 19 × 13 cm) with free access to food and water and maintained under controlled temperature (22 ± 1°C) and 12:12 light/dark cycle (lights on at 7:00 am). All experiments were conducted during the light phase. All procedures were approved by the Ethical Committee for Animal Use at UNIFESP (CEUA # 0074/12 and #2406280214).

### 2.2. Drugs

Nicotine 99% (Sigma, St Louis, MO) was diluted in saline (0.9% NaCl) and subcutaneously administered (doses of 0.1; 0.4 or 1.0 mg/kg, s.c.). The choice of nicotine doses was based in literature data [35–37], and selected doses were further tested in mice, after acute and intermittent treatment, in Experiment 1 (see Section 2.5.1).

Methamphetamine dose was based on data from previous studies in our laboratory, showing clear stimulant effects after 1.0 mg/kg [38, 39]. Methamphetamine was donated by the Federal Police (São Paulo, Brazil), diluted in saline and administered intraperitoneally. Drug treatments and saline were administered in a volume of 10 ml/kg body weight.

### 2.3. Locomotor Activity Test

Locomotor activity was assessed by automated activity monitoring chambers (Opto M3, Columbus Instruments, Columbus, Ohio). The chambers were 47.5 cm high x 25.7 cm long x 20.5 cm wide and contained 16 pairs of photoelectric beams in the horizontal axis. The subsequent interruption of two beams was recorded as one unit of locomotor activity. Locomotor activity of mice was recorded for 30 minutes immediately after drug administration during activity test days.

### 2.4. Social Defeat Stress

The subjects were allocated into control or defeat stress groups. Mice in stress groups (intruders) were defeated by another conspecific male aggressor (resident), which was previously housed with a receptive female and trained to present reliable levels of aggressive behavior. The detailed social defeat protocol was previously described by Favoretto et al., 2017 [40].

Training of residents consisted in the confrontation of an unfamiliar conspecific male, introduced into the resident's home cage (3 sessions/week, during 3-4 weeks), until the resident presented stability in aggressive behavior (15% variation in attack bites within 3 successive confrontations).

One episode of social defeat consisted of 3 phases [41]: (1) Initiation phase (5 minutes): after the removal of the female, the intruder was introduced into the home cage of the aggressive resident, separated by a perforated acrylic partition, which allowed auditory, olfactory, and visual contact between the animals, but no physical confrontation. (2) Defeat phase: the acrylic wall was removed and the resident was able to persecute, threaten, and attack the intruder. The defeat phase lasted up to five minutes, being interrupted earlier if the intruder presented submissive posture for 4 consecutive seconds, or any sign of injury. (3) Threat phase: resident and intruder were again separated by a perforated acrylic wall for five minutes (episodic defeat), and the intruder was then returned to its home cage until the next defeat, 24 h later. In the protocol for continuous defeat, the defeated mouse was kept in cohabitation and sensorial contact with the aggressive resident for 24 hours until the next defeat, with free access to food and water, as described by Golden et al. [42].

Both protocols of social defeat occurred for 10 days, with one daily confrontation. Average number of attack bites received by defeated mice in each experiment is shown in Table 1. Aggressive residents were rotated, so that each day a different aggressor defeated the intruder, in order to avoid habituation. Control mice for episodic stress were kept isolated and undisturbed in their home cages, being handled every two days for weighing and cleaning purposes. For the continuous stress protocol, controls were kept for 10 days in cohabitation with another control animal, using the same acrylic partition that was used for the defeats. Controls for the continuous stress had their housing partners rotated every day, as described by Golden et al., 2011 [42]. At the end of the 10-day stress protocol, all subjects were returned to their individual home cages.

### 2.5. Experimental Procedures

#### 2.5.1. Experiment 1: Characterization of Nicotine-Induced Psychomotor Effects

Prior to any manipulation, mice were exposed for 30 minutes to the locomotor activity cage (novelty test) and then were distributed into four groups with homogeneous averages for body weight and baseline locomotor activity. During the next thirteen days, mice received daily injections of saline (control group, n=10) or different doses of nicotine (0.1 (n=10); 0.4 (n=11) or 1.0 (n=10) mg/kg) [35]. Locomotor activity was tested for 30 minutes immediately after the saline or nicotine injection on days 1, 4, 7, 10, and 13. The locomotor challenges were performed 48 hours after the end of intermittent treatment. Mice were exposed to a saline challenge on day 15, a 0.1 mg/kg nicotine challenge on day 17, and a 0.4 mg/kg nicotine challenge on day 19. Locomotor activity was recorded for 30 minutes after each injection. Since the effects of intermittent nicotine treatment may be observed even after 21 days of withdrawal [35, 36], another nicotine 0.4 mg/kg challenge was conducted on day 36 (after 17 days of nicotine withdrawal) (Figure 1(a)).

#### 2.5.2. Experiment 2: Consequences of Two Social Defeat Protocols (Episodic or Continuous) on the Locomotor Effects of Nicotine

Similarly to the previous experiment, different batches of mice were weighed and exposed for 30 minutes of novelty test at the locomotor activity cage and then were homogeneously distributed into two groups based on their weight and locomotor activity. For each social defeat procedure (episodic or continuous), one set of control and stress groups were allocated. Animals were then exposed to social defeat stress for 10 days, as shown in the experimental timeline (Figure 1(b)). Three hours after the final episodic defeat or three hours after the end of the cohabitation period (for continuous defeat stress), animals were tested in locomotor activity cages after receiving a saline injection (saline challenge). Twenty-four hours later, mice were tested after a nicotine injection (nicotine challenge, 0.1 mg/kg). The saline and nicotine challenges were performed again at 9 and 10 days, respectively, after the end of social defeat protocol. Additionally, two days after the final nicotine challenge, mice were exposed to a methamphetamine challenge (1.0 mg/kg, i.p.) in order to check for their ability to present drug-induced locomotor stimulation.

### 2.6. Data Analysis

All data are presented as means ± standard error (SE). Locomotor activity (as assessed by number of beam breaks) was analyzed with two-way Analysis of Variance (ANOVA), using groups as one factor, and tests or challenges as the second factor (with repeated measures). Further one-way ANOVAs were used to detect possible group effects on separate test days. Newman-Keuls tests for multiple comparisons were used for post hoc analysis when the ANOVA detected significant effects. The level of significance was set to 5%.

## 3. Results

### 3.1. Experiment 1: Characterization of Nicotine-Induced Psychomotor Effects

A one-way ANOVA showed no preexisting group differences between during the novelty tests (F(3,33)=1.23, p=0.31).

A repeated measure ANOVA compared locomotor responses of control and nicotine-treated groups over the course of the 13-day treatment. Significant effects were detected for Group (F(3,36)=9.20, p<0.001), Locomotor tests (F(4,144)=39.85, p<0.001), and Group versus Test Interaction (F(12,144)=3.86, p<0.001). Post hoc analysis of the Group effect showed that group treated with 1.0 mg/kg nicotine was different from all other groups (p<0.05). On test day 13, post hoc analysis of the Interaction revealed that all groups showed increased locomotor activity relative to test day 1, except for mice treated with 1.0 mg/kg nicotine, which displayed significant suppression of activity relative to all other groups.

One-way ANOVAs for each test day revealed significant additional group differences (Figure 2). On the 1st test day (F(3, 36)=10.35, p<0.001), mice treated with 0.4 or 1.0 mg/kg of nicotine showed reduced locomotor activity relative to controls or 0.1 mg/kg nicotine group (p<0.05). On the 2nd test day (F(3, 36)=5.23, p=0,004) only the group injected with 1.0 mg/kg of nicotine showed reduced locomotor activity relative to controls and 0.1 mg/kg groups (p<0.05). On the 3rd test (F(3, 36)=5.85, p=0.002), mice treated with 1.0 mg/kg of nicotine displayed significantly lower activity from all other groups (p<0.05). On the 4th test day (F(3, 36)=11.67, p<0.001), mice treated with 0.1 mg/kg nicotine showed increased activity (p<0.05), and those treated with 1.0 mg/kg of nicotine showed reduced locomotor activity (p<0.001) relative to the other two groups (controls and 0.4 mg/kg nicotine group). On the 5th test day (F(3, 36)=8.23, p<0.001), only the group injected with the higher 1.0 mg/kg nicotine dose showed reduced locomotor activity relative to all the others groups (p<0.001).

To assess the expression of the nicotine psychomotor effects, controls and nicotine-treated groups were challenged with further saline and nicotine locomotor tests (Figure 3). A repeated measure ANOVA was conducted comparing control and nicotine groups during the challenges. Significant effects were detected for Group (F(3,36)=3.14, p=0.04), Challenges (F(3,108)=53.51, p<0.001), and Group versus Challenge (F(9,108)=5.15, p<0.001). Control mice showed reduced activity when challenged with a 0.4 mg/kg nicotine dose (p<0.001), and so did mice previously treated with the lower 0.1 mg/kg nicotine dose (p<0.001). Mice with a history of treatment with 0.4 mg/kg nicotine expressed tolerance to its psychomotor suppression effect (p<0.05), observed during the short-term challenge with the same dose. However, during the long-term nicotine challenge (0.4 mg/kg), nicotine reduced activity of all groups when compared to the saline challenge, except for the group with a history of intermittent treatment with the higher 1.0 mg/kg nicotine dose.

Separate one-way ANOVAs for each challenge revealed significant additional group differences. During the saline challenge (F(3, 36)=4.64, p=0.008), the group pretreated with the higher 1.0 mg/kg nicotine dose showed lower locomotor activity than all other groups (p<0.05). On the 0.1 mg/kg nicotine challenge (F(3, 36)=3.3991, p=0.028), the group pretreated with 1.0 mg/kg nicotine dose showed reduced locomotor activity relative to other nicotine-treated groups (p<0.05), but not different from control group (p=0.3). On the short-term 0.4 mg/kg nicotine challenge (F(3, 36)=3.6783, p=0.02), only the group pretreated with nicotine 0.4 mg/kg showed higher locomotor activity levels relative to controls (p=0.01). On the long-term 0.4 mg/kg nicotine challenge F(3, 36)=3.0325, p=0.042) the group pretreated with 0.4 mg/kg of nicotine showed higher activity response to nicotine relative to controls (p=0.03).

### 3.2. Experiment 2: Consequences of Two Social Defeat Protocols (Episodic or Continuous) on the Locomotor Effects of Nicotine

A one-way ANOVA showed no preexisting differences during the novelty tests neither between episodic stress group and its controls (F(1, 16)=0.16, p=0.69), nor between continuous defeated mice and their controls (F(1, 14)=0.03, p=0.88).

A repeated measure ANOVA comparing episodic defeat stress and its controls during the locomotor tests (nicotine/saline) (Figure 4) revealed a significant interaction between stress and locomotor tests (F(3,48)=3.39, p=0.025) and also a significant test effect (F(3,48)=8.44, p<0.001) (Figure 4(a)). Post hoc analysis of the interaction revealed no significant locomotor effects of nicotine in the episodic stress group, relative to the locomotor response to saline, whether short-term or long term. However, the locomotor response to long-term nicotine/saline challenges was higher than the short-term tests (p<0.05), suggesting short-term stress-induced locomotor suppression. Within controls, a blunted locomotor response to the first nicotine challenge was observed, compared to the first saline challenge (p<0.05). This sedative locomotor effect of nicotine was no longer presented in the long-term nicotine challenge. There were no group differences (stress versus control) in any test. Time course of nicotine-induced locomotor effects during the short-term and long-term challenges is shown in Figures 4(b) and 4(c), respectively. No significant group effect or group X time interaction was obtained for the time course analysis.

For the continuous defeat protocol (Figure 5), a repeated measure ANOVA revealed a significant effect for stress (F(1,14)=18.6, p=0.001) and locomotor tests (F(3,42)=5.8, p=0.002), with a significant interaction between factors (F(3,42)=4.13, p=0.012) (Figure 5(a)). Post hoc analysis of the interaction revealed group differences during both short-term saline and nicotine tests, when continuous defeat stress group presented suppressed locomotor activity relative to controls (p<0.05). No group differences were observed during the long-term tests. Within-group comparisons for the continuous stress group suggest a trend for additive effects of nicotine on stress-induced short-term suppression of locomotor activity (p=0.06). Furthermore, no further locomotor suppression was observed during the long-term nicotine challenge, in which stressed mice showed higher activity relative to the short-term nicotine test (p<0.05), suggesting the occurrence of tolerance to nicotine locomotor effects. In the control group, suppression of locomotor activity was observed after the first nicotine challenge, relative to the saline test (p<0.05). Nicotine-induced suppression was no longer observed in the long-term test for controls. Time course of nicotine-induced locomotor effects during the short-term and long-term challenges is shown in Figures 5(b) and 5(c), respectively. Statistical results confirm the overall analysis of collapsed data (Figure 5(a)), with no further group X time interaction.

To assess whether previously stressed mice were capable of presenting psychomotor stimulation, we evaluated their locomotor response to a psychostimulant drug, methamphetamine (1.0 mg/kg, i.p.), two days after the final nicotine test (Figure 6). These data were compared with the response to the second saline challenge. Repeated measures ANOVA detected a significant challenge effect (F(1,16)=21.35, p<0.001) for episodic defeat (Figure 6(a)). In the episodic defeat protocol, methamphetamine induced significant hyperactivity in both control and stress groups (p<0.05). Time course of methamphetamine-induced locomotor effects is depicted in Figure 6(b) for episodic stress and respective controls. For the continuous defeat protocol (Figure 6(c)), repeated measures ANOVA detected significant challenge effect (F(1,14)=13.52, p=0.002). Methamphetamine administration induced hyperactivity in the control group (p<0.05), with a trend for stimulation in the stress group (p=0.068).

## 4. Discussion

To our knowledge, this is the first study to systematically characterize the psychomotor effects of 3 different doses of nicotine in mice (0.1; 0.4 and 1.0 mg/kg), considering acute nicotine effects; effects during repeated, intermittent nicotine administration; and the expression of nicotine psychomotor effects after short and long periods of withdrawal. This is also the first study to systematically address the impact of two types of social defeat stress (episodic and continuous) on nicotine-induced psychomotor effects.

### 4.1. Characterization of Nicotine-Induced Psychomotor Effects

Concerning nicotine-induced locomotor effects, nicotine promoted dose-dependent and time-dependent (acute versus chronic) effects. Acute administration of 0.4 and 1.0 mg/kg of nicotine promoted locomotor suppression, while the lower nicotine dose promoted no significant psychomotor effects. After four days of intermittent nicotine administration, the locomotor activity of mice treated with 0.4 mg/kg was no longer different from the control group, suggesting the development of tolerance to nicotine-induced suppression, as reported by Domino (2001) in Sprague Dawley rats [36]. After ten days of repeated nicotine administration, the group treated with 1.0 mg/kg continued presenting robust locomotor suppression, while the group treated with 0.4 mg/kg continued to show similar levels of locomotor activity as the saline-treated group. On test day 10, mice repeatedly treated with the lower dose (0.1 mg/kg) of nicotine showed significant higher locomotor activity relative to all other groups, which could indicate the development of locomotor sensitization. However, this sensitized effect was not sustained, and statistical differences were no longer observed on test day 13. On day 13, the only group difference concerned the group treated with the high nicotine dose (1.0 mg/kg), which continued to present locomotor suppression.

The expression of behavioral effects to saline/nicotine challenges started after two days of withdrawal from repeated nicotine administration. During the saline challenge (day 15), the group pretreated with 1.0 mg/kg of nicotine still presented lower locomotor activity than the other groups, and such suppressed activity was also observed during the first nicotine 0.1 mg/kg challenge, on day 17. Suppressed locomotor activity after saline or after the low nicotine dose may be due to a contextual conditioning effect induced by the high 1.0 mg/kg nicotine dose [9], since neither the saline nor the lower dose of nicotine should induce locomotor suppression. Thus, our data suggest that previous exposure to a high nicotine dose may induce conditioned suppression of locomotor activity when mice are challenged in the same testing environment where they experienced the effects of a high dose of nicotine.

Additionally, mice were challenged with the intermediate dose of nicotine (0.4 mg/kg) on days 19 and 36, representing short- and long-term withdrawal periods from repeated, intermittent nicotine treatment. During the short-term 0.4 mg/kg nicotine challenge, saline-controls showed the expected locomotor suppression. Mice previously treated with 0.4 mg/kg nicotine showed significantly higher locomotor activity relative to the saline group, suggesting tolerance to nicotine-induced locomotor suppression. Such tolerance was also observed during the long-term challenge with the intermediate nicotine dose, in the group of mice pretreated with the same 0.4 mg/kg dose.

In summary, the dose of 0.1 mg/kg nicotine showed a trend to induce stimulant effects after repeated, intermittent nicotine administration, with no acute locomotor effects in naïve mice. The dose of 0.4 mg/kg nicotine induced acute locomotor suppression with tolerance after repeated administration, and the dose of 1.0 mg/kg induced long lasting locomotor suppression. Since our hypothesis was that exposure to episodic, but not continuous, defeat stress would facilitate and/or potentiate the locomotor stimulant response to nicotine, in the second experiment we only used the lower dose of nicotine (0.1 mg/kg) to test the animals after the social defeat protocols.

### 4.2. Interactions of Social Defeat Stress and Psychomotor Effects of Nicotine

Continuous and episodic social defeat stress induced suppression of locomotor activity in the short-term (24h after stress), which was no longer observed 9 days after the end of social defeat protocol. Nicotine potentiated short-term locomotor suppression induced by continuous, but not episodic, social stress. However, when mice were tested 10 days after the continuous defeat stress protocol, there was tolerance to the sedative effects of nicotine in continuously stressed mice.

Social defeat stress has been reported to suppress locomotor activity [43–45], as we also found in our study. However, this was an effect with limited duration, only observed during short-term locomotor challenges (within 24-h after repeated stress), but not during long-term challenges (9-10 days after repeated stress). In our studies, the short-term suppression of activity after social stress was observed after both episodic and continuous defeat. Miczek et al., 2011 [18], showed that chronic continuous, but not episodic, defeat stress reduced exploratory behavior in the open field test within a few hours after defeat. Similarly to our study, neither episodic nor continuous defeat affected the locomotor response to a saline challenge 10 days after end of the stress protocol [18]. The absence of short-term suppressive effects after episodic defeats in Miczek et al., 2011 [18], may be due to protocol differences, since the episodic stress protocol consisted of four defeat episodes separated by 72-hour intervals (4 defeats in 10 days), while the continuous protocol comprised five defeats/week, during 5 weeks [18].

In mice with a history of episodic defeats, a low nicotine dose did not produce any locomotor effects. On the other hand, nicotine seems to potentiate the short-term locomotor suppression in continuously stressed group, an effect no longer observed during the long-term nicotine challenge, possibly due to the development of tolerance to nicotine psychomotor effects. In our laboratory, a separate study verified the impact of episodic versus continuous defeat stress on nicotine effects, using the intermediate dose of 0.4 mg/kg, with slightly different procedures for locomotor testing (data not published). Significant suppression of locomotor activity was found in both controls and stressed mice when challenged with 0.4 mg/kg nicotine, both in short-term and long-term nicotine challenges (24h or 10 days after stress). Altogether, our current study and these data suggest a dose-dependent relationship between stress and nicotine, in which a significant impact of social defeat stress on nicotine-related effects was only observed after a low nicotine dose.

Our results suggest that the consequences of stress exposure on nicotine locomotor effects may be different for social defeat stress when compared to other types of stressors. For example, Cruz et al., 2008 [21], found that chronic restraint stress enhanced the stimulant effect of nicotine in rats, although another study failed to detect a significant impact after similar stress procedure [46]. Leão et al., 2012 [23], found that exposure to chronic variable stress increased nicotine-induced locomotor activity. Since these studies were carried out in rats, there is also a possibility of species differences (rats versus mice) in sensitivity to repeated stress and/or to nicotine itself.

Furthermore, the impact of social defeat stress on drug effects may be dependent on the drug tested. For example, there is evidence that social defeat stress in mice promotes a sensitized response to an amphetamine challenge [47], but locomotor response to ethanol was unaffected after repeated episodic defeats [34]. In our laboratory, we observe that mice with a history of continuous defeat stress fail to show locomotor stimulation after an ethanol challenge [48], while exposure to episodic defeats had no impact on ethanol's effects (Macedo et al., unpublished). In the present study, we also observed that even 12 days after the stress protocol, continuous but not episodic defeat seems to attenuate the stimulant effect of methamphetamine. Thus, different consequences of social defeat may be observed according to the defeat protocol (episodic versus continuous) and to the drug tested. In this study, continuous defeat stress further aggravated nicotine-induced suppression of locomotor activity within 24 h after stress and also attenuated methamphetamine-induced hyperactivity in the long term.

While in our study the exposure to stress and nicotine occurred in separate temporal phases of the protocol, other studies have evaluated the consequences of concomitant exposure to stressors and nicotine. For example, Kita et al., 1999 [49] found that rats receiving nicotine immediately after each session of chronic psychological stress (witnessing other rats receiving footshock stress) presented enhanced nicotine-induced sensitization at 5 and 10 days of the combined treatment. On the other hand, Harris et al., 2014 [50], found that simultaneous exposure to nicotine during chronic restraint stress prevented the short-term locomotor suppression induced by the stress protocol, although no long-term effects on nicotine locomotor response were observed (see also [46]). Thus, not only the type of stressor, but also the timing of nicotine and stress exposures may be critical to determine the outcomes of stress exposure on nicotine-induced locomotor effects.

Future studies should verify conditions in which social defeat stress may further interfere with nicotine effects, whether using different doses or changing the timing of stress exposure in relation to nicotine administration.

In summary, this study shows dose-dependent and time-dependent effects of nicotine on locomotor behavior of mice. A lower nicotine dose tended to induce locomotor stimulation after repeated, intermittent treatment, while an intermediate dose produced initial locomotor suppression to which tolerance developed. The highest nicotine dose promoted consistent and robust locomotor suppression that was not changed over time and seems to produce conditioned locomotor suppression. Both episodic and continuous defeat stress protocols induced short-term locomotor suppression (24h after stress), which was further suppressed by a low dose of nicotine only in mice exposed to continuous defeat stress. Furthermore, while exposure to social stress failed to affect long-term locomotor response to nicotine challenge, mice exposed to continuous defeats showed a reduced stimulant response to methamphetamine, 12 days after termination of stress. Thus, continuous social defeat stress facilitates nicotine-induced locomotor suppression shortly after stress, and reduces methamphetamine-induced stimulation in the long term.

## Figures and Tables

**Figure 1:** Experimental design for Experiment 1 (a), characterization of nicotine-induced psychomotor effects, and Experiment 2 (b), consequences of social defeat on the psychomotor effects of nicotine. (a) Four groups of mice were daily injected with saline, 0.1, 0.4, or 1.0 mg/kg (s.c.) of nicotine for 13 days, during which 5 locomotor test days were carried out. Additional saline and nicotine challenges were scheduled after short- and long-term withdrawal from intermittent nicotine treatment. (b) One group of mice underwent 10 days of episodic stress (and its corresponding control group), and another group underwent 10 days of continuous social stress (with its respective control group). After termination of chronic stress, mice were tested for locomotor activity after saline and nicotine (0.1 mg/kg, s.c.) challenges, shortly after stress (~1 day) or after ~10 days. Locomotor activity was also tested after a methamphetamine challenge (1.0 mg/kg, i.p.), on day 22.

**Figure 2:** Locomotor activity of mice in response to daily saline or nicotine (0.1, 0.4, or 1.0 mg/kg, s.c.) treatment. Locomotor tests were carried out on treatment days 1, 4, 7, 10, and 13, immediately after injection, and activity was recorded during 30 minutes. *∗* Different from the control group. In all cases, p<0.05.

**Figure 3:** Locomotor activity in response to saline and nicotine (0.1 and 0.4 mg/kg, s.c.) challenges, in mice previously exposed to 13-day treatment with different nicotine doses (0.1, 0.4, or 1.0 mg/kg, daily). Short-term challenges were carried out within 2, 4 and 6 days after the end of the intermittent treatment, while long-term nicotine challenge was carried out 17 days after the last short-term challenge. *∗*Different from the control group on the same challenge day; #within-group difference relative to the saline challenge. In all cases, p<0.05.

**Figure 4:** (a) Locomotor activity in response to saline and nicotine (0.1 mg/kg, s.c.) challenges, in mice previously exposed to repeated episodic defeat stress protocol. Short-term challenges were carried out within 3 h (saline) and 24 h (nicotine) of the final defeat, while long-term challenges were carried out after 9 and 10 days after defeat. (b) and (c) show the time course of nicotine-induced locomotor effects in 5-min bins, during short-term (b) and long-term (c) challenges. +Difference between saline and nicotine challenges (within-group comparison). #Difference between respective short- and long-term challenges. In all cases, p<0.05.

**Figure 5:** (a) Locomotor activity in response to saline and nicotine (0.1 mg/kg, s.c.) challenges, in mice previously exposed to repeated continuous defeat stress protocol. Short-term challenges were carried out within 3 h (saline) and 24 h (nicotine) of the final defeat, while long-term challenges were carried out after 9 and 10 days after defeat. (b) and (c) show the time course of nicotine-induced locomotor effects in 5-min bins, during short-term (b) and long-term (c) challenges. *∗*Difference between control and stressed group in the same test; +Difference between related saline and nicotine challenges (within-group comparison). #Difference between related short- and long-term challenges. In all cases, p<0.05.

**Figure 6:** Locomotor activity in response to methamphetamine (1.0 mg/kg, i.p.), 2 days after the long-term nicotine challenge (12 days after stress), in (a) mice previously exposed to episodic defeat protocol; (c) mice previously exposed to continuous defeat stress protocol. Figures (b) and (d) show the time course of locomotor response to methamphetamine in mice exposed to episodic and continuous protocols, respectively. +Difference between long-term saline and methamphetamine challenges (within-group comparison). In all cases, p<0.05.

**Table 1:** Average number of bites (mean ± SE) received by defeated mice undergoing repeated episodic defeats or continuous defeat stress.

	Bites/Defeat day (Mean ± SE)									
Group	D1	D2	D3	D4	D5	D6	D7	D8	D9	D10
Episodic Stress (n=8)	12 ± 2	19 ± 3	15 ± 3	18 ± 2	15 ± 3	21 ± 1	10 ± 2	16 ± 3	10 ± 2	13 ± 2
Continuous Stress (n=8)	21 ± 3	23 ± 3	13 ± 2	15 ± 2	12 ± 2	12 ± 2	8 ± 1	13 ± 2	7 ± 1	8 ± 1

## Data Availability

The data used to support the findings of this study are available from the corresponding author upon request.
